The article "Robust Parameter Design for Cyclone System Based on Dual-Response Surface Method and Multiobjective Genetic Algorithm" was published in 2022. Journal: Comput Intell Neurosci.

# Robust Parameter Design for Cyclone System Based on Dual-Response Surface Method and Multiobjective Genetic Algorithm

**DOI:** 10.1155/2022/5884868

**Published:** 2022-06-18

**Authors:** Fusheng Luo, Xianhui Yin, Zhanwen Niu

**Affiliations:** ^1^College of Management and Economics, Tianjin University, Tianjin 300072, China; ^2^School of Management, Hainan University, Haikou, Hainan 570228, China; ^3^College of Quality and Standardization, Qindao University, Qindao, Shandong 266071, China

## Abstract

To realize the predictive control of coal preparation quality and ensure that the quality of washing products is close to the minimum coal quality requirement of coal blending to the greatest extent is one of the important means to maximize production and maintain the interests of customers and enterprises. Therefore, the feasibility of introducing the double response surface method and multiobjective genetic algorithm to solve the aforementioned problems is further discussed. By selecting the controllable factors and noise factors affecting the output and determining their respective value levels, the product table method is used to design the robust parameter design test, and the experimental results are obtained, according to the experimental data, the second-order polynomial model of the mean and standard deviation of each response characteristic is established, and the effectiveness of the model is analyzed. Then, the double-response optimization function of each response characteristic is established according to the type of response characteristic. Finally, the corresponding parameter values are solved by multiobjective genetic algorithm. The internal and external surface method is used to design and run 60 tests. Through optimization analysis, the robust parameter settings are 150.68 kpa, 0.18143.73 kpa, and 30%, and the optimal output is ash 8.499%, which yields 69.54%, meeting the requirements of stakeholders. Moreover, compared with the traditional optimization design method, the superiority of the proposed method is verified, which shows that this method is conducive to the transformation of the coal preparation plant from fire-fighting quality management to preventive quality management and provides support for the accurate control and systematic management of the production process of the coal preparation plant.

## 1. Introduction

Coal preparation is the main technological process for the value-added of coal products. It is the key link for coal enterprises to identify customer needs, meet customer needs, and create enterprise value. Therefore, the qualification and stability of product quality and the washing rate in the coal preparation process directly affect the coal preparation effect. If the quality of washing products fluctuates greatly or is out of control, it will not only bring technical problems to the subsequent coal blending and affect the interests of customers but also cause enterprises to pursue too high quality and reduce the washing rate to meet the requirements of coal blending, so as to bring benefit losses to enterprises. In order to ensure the stability of coal preparation product quality and maximize the washing rate, experts and scholars at home and abroad have conducted a lot of research. As the coal preparation process is the fundamental reason affecting the washing effect, the process method has always been the focus of research. At present, the most commonly used coal preparation processes at home and abroad are heavy medium coal preparation and flotation. As the flotation technology is only suitable for coal slime with small particle size, its application scope is limited. In contrast, heavy medium coal preparation has the advantages of high separation accuracy and strong adaptability to raw coal and has gradually become the mainstream coal preparation technology at present [1]. Therefore, this study selects the heavy medium coal preparation plant as the research object and discusses the method to realize multiobjective stable output under the condition of determining the coal preparation process. In addition to process methods, some experts and scholars have studied the methods to ensure coal quality and washout rate from the perspective of management and evaluation. For example, Li [2] put forward 11 suggestions to ensure coal quality, and Gong and Xu [3] studied the performance evaluation method of quality management of coal preparation plant, both of which have played a certain role in promoting the guarantee of coal quality and the improvement of benefits. Other scholars have studied the setting of process parameters in the production process, such as feeding mode and feeding pressure [4–6], established the mapping relationship between process parameters and quality characteristics through historical data, and determined the value range of each parameter. Other scholars have studied the application of quality management tools in the coal preparation plant, such as Elevli [7] studied the application of control chart in the coal preparation plant and realized the abnormal monitoring and control of coal preparation product quality. Xi Jin et al. [8] used the nonlinear regression method to study the optimal combination of various parameters in the coal blending link, which provides a basis for the production control and optimization of coal blending. However, the existing research on coal quality and yield control methods in coal preparation process mainly focuses on postdetection. Even the research on parameter optimization is also the optimization of single-response characteristics, does not consider the common optimization problem between quality and efficiency at the same time, and ignores the influence of noise factors on the robust output of production system in the optimization process. In addition, the existing studies mainly focus on the independent optimization of single factors and lack of systematic research on the impact of coal preparation production system on coal quality and yield. As the heavy medium coal preparation is a huge and complex production system, involving hundreds of equipment and thousands of processes, if the whole system is optimized and analyzed, a large amount of data needs to be collected, even a large number of tests need to be carried out, and the research cost is too high. Therefore, the key subsystems of the whole production system are selected for analysis. The principle of subsystem optimization indirectly reflects the process of realizing the optimal output of the whole production system. As the core-processing process in the production process of heavy medium coal preparation, cyclone separation is the key control link to achieve stable quality and maximum yield of heavy medium coal preparation. It is also the key subsystem in the production system of heavy medium coal preparation. Therefore, the robust parameter design of multiobjective-oriented cyclone production system has become a problem worthy of study. Experts and scholars at home and abroad have done a lot of research on the optimal design of hydrocyclone. Sun et al. [9] and Liu et al. [10], respectively, used the grey correlation method and RSM (Reynolds stress model) to study the setting of relevant parameters such as volume concentration and flow field of cyclone in heavy medium coal preparation plant. Azizi et al. [11] studied the application of Plackett Burman method in identifying key factors of coal preparation and achieved remarkable results. Chen et al. [12] and Zhang Guo et al. [13] studied the method of parameter control database and linear regression to realize the identification and automatic control of the relationship between parameters *s*. In addition, many scholars have studied the online optimization and control method of heavy medium coal preparation, the optimal method of coal preparation process design, the optimization method of process yield, and the optimal realization method of cost and quality. [14–20].

The article "Robust Parameter Design for Cyclone System Based on Dual-Response Surface Method and Multiobjective Genetic Algorithm" was published in 2022. Journal: Comput Intell Neurosci.

However, the aforementioned optimization methods have the following shortcomings: (1) the established optimization function is a function of single-response characteristics, without considering the multiobjective optimization of quality and efficiency; (2) the fitting model established by Plackett Burman experimental design method does not consider the interaction between controllable factors; (3) the existing optimization design methods do not consider the influence of noise on the system output; (4) many existing optimization model data basically come from the historical data of field production, so the representativeness of analysis samples and the effectiveness of data seriously restrict the accuracy of the model. The shortcomings of these studies show that the existing methods cannot determine the value of the best operating parameters that can ensure the robust output of the system under the multiobjective guidance. The study of a system parameter setting is essentially a process of changing the concept of quality management, that is, from the original fire-fighting and passive quality management to preventive and autonomous management. In order to achieve this purpose, many advanced methods have studied by experts and scholars, such as Cheng and Pan [21], Lv et al. [22], and Yan [23], have studied the application of DOE method in the specific production process of machinery manufacturing industry. The significant factors affecting specific output are identified, the optimal parameter setting is confirmed, and the output performance index is greatly improved. Lecureux et al. [24] studied the influence of specific influencing factors on electromagnetic sunscreen through DOE technology, providing data support for the optimization of electromagnetic sunscreen production system. Smith et al. [25] and Moscynski [26] studied the application of DOE technology and method in aerospace field. In terms of precision analysis and control, Yoon et al. [27] applied this method to the parameter optimization analysis of the robot foot control system to realize the optimal parameter configuration of the overall system with multiple inputs and outputs. Doe has also been gradually studied and applied in the fields of chemical industry, service industry, performance evaluation, and cost management [28–30]. For the influence of noise factors on system output, Taguchi [31], a Japanese scholar, first systematically proposed the concept of robust parameter design, which was realized by internal and external table design method and signal-to-noise ratio analysis. Although this method has been widely used, it is questioned by Miller [32], Montgomery [33], Tsui [34], and other scholars because it does not consider the interaction between factors, the experiment is lack of sequence, and the SNR index is unreasonable. As an improvement, Vining and Myers [35, 36] expressed the RPD problem as a constrained optimization problem and proposed dual-response surface methodology (DRSM) to solve this problem. Its basic idea is to fit the two response surfaces of the process mean and variance respectively, and then minimize the variance with the mean target value as the constraint, so as to improve the robustness of the process. For example, Zhao et al. [37] studied the robust parameter design of double-response surface method in the process of solder paste printing, which improved the quality of solder paste thickness and reduced the volatility. He et al. [38] took the tire product design of a rubber company in Tianjin as the object, optimized an important quality feature (rubber hardness) in the tire production process using the double-response surface method and designed the test design software according to the double-response surface method. The test design results found the ratio conditions to achieve the rubber hardness target and reduce the hardness variation. By adjusting the combination of controllable factors, the double-response surface reduces the sensitivity of the system to noise factors and ensures the robustness of the system. However, the existing double-response surface analysis mainly solves the robust parameter design problem of single-response characteristics, and the optimization of production system includes two dimensions of quality and efficiency and multiple-response characteristics.

The article "Robust Parameter Design for Cyclone System Based on Dual-Response Surface Method and Multiobjective Genetic Algorithm" was published in 2022. Journal: Comput Intell Neurosci.

Therefore, the main contribution of this research is to explore the method of robust parameter design of hydrocyclone production system under the condition of multiresponse characteristics. First, the double-response surface method for the response characteristics of quality and efficiency is studied, and the double-response function of each response characteristic is established. Then the multiobjective genetic algorithm is used to solve the evaluation problem of multiobjective optimization function under constraints, and finally, the robust parameter values under multiobjective conditions are obtained. The superiority of the proposed method is illustrated by comparing the traditional satisfaction function method with the gradient descent method.

Based on the aforementioned discussions, the main contributions are given as follows:

1. In this paper, the dual-response surface method is applied to the robust parameter design of cyclone system for the first time, which provides a new idea for the follow-up research.
2. For the parameters that have been estimated, the optimization algorithm is used to optimize, so that more accurate and fine results can be obtained

The article "Robust Parameter Design for Cyclone System Based on Dual-Response Surface Method and Multiobjective Genetic Algorithm" was published in 2022. Journal: Comput Intell Neurosci.

## 2. Double-Response Surface Method

Suppose the response variable is *Y* and the controllable variable is *X*_1_, *X*_2_, and *X*_*K*_, repeat the measurement on the response variable *Y*, and calculate its mean and standard deviation. Taking the mean and standard deviation of the response as output variables, Vining and Myers fit the second-order polynomial model respectively:

(1) $$\begin{array}{c} \omega_{u}\left(x\right)=\beta_{0}+\sum_{i=1}^{k}\beta_{i}x_{i}+\sum_{i=1}^{k}\beta_{ii}x_{i}^{2}+\sum \sum_{i<j}^{k}\beta_{ij}x_{i}x_{j}+\varepsilon_{u},\\ \omega_{\sigma }\left(x\right)=\gamma_{0}+\sum_{i=1}^{k}\gamma_{i}x_{i}+\sum_{i=1}^{k}\gamma_{ii}x_{i}^{2}+\sum \sum_{i<j}^{k}\gamma_{ij}x_{i}x_{j}+\varepsilon_{\sigma }. \end{array}$$

As two models are used to optimize the mean and standard deviation, how to select the optimization function to optimize the mean and standard deviation at the same time is a problem that engineers and technicians must solve. For example, when Vining and Myers optimize the quality characteristics of the target type, the optimization method they select is as follows:

(2) minω,σs.t.ωu=τ,L≤xi≤U, i=1,2,…k..

where *ω* is the target value, and *l* and *u* are the boundary of *x* value. Formula (2) can also be transformed into

(3) $$\begin{array}{c} \left\{\begin{array}{cc} \min & F\left(x\right)=\omega_{\sigma }^{2}+{\left(\omega_{u}-\tau \right)}^{2},\\ s.t. & L\leq x_{i}\leq U,i=1,2,\ldots k. \end{array}\right. \end{array}$$

## 3. Multiobjective Genetic Algorithm

The multiobjective optimization problem can be described as follows:

(4) $$\begin{array}{c} \left\{\begin{array}{cc} \min & \left[F_{1}\left(x\right),F_{2}\left(x\right),F_{3}\left(x\right)\right],\\ \mathrm{s.t}. & \left\{\begin{array}{c} lb\leq x\leq ub,\\ \text{Aeq}*x=\text{beq}\\ A*x\leq b, \end{array},\right. \end{array}\right. \end{array}$$

where min[*F*_1_(*x*), *F*_2_(*x*),…, *F*_*m*_(*x*)] is the objective function to be optimized; *X* is the variable to be optimized; *lb* and *ub* are lower bound and upper bound of variables, respectively; Aeq*∗x*=beq is the equality constraint of *X*; *A∗x* ≤ *b* and *lb* ≤ *x* ≤ *ub* are the inequality constraints for *X*.

Since the objective functions may be contradictory, that is, the improvement of one objective function may require the reduction of another objective function as a cost. As shown in Figure 1, *A*1 < *B*1 and *A*2 > *B*2 call such solutions *A* and *B* noninferior solutions, or Pareto optimal solutions. The purpose of multiobjective optimization algorithm is to find these optimal solutions.

At present, there are many multiobjective optimization algorithms. Kalyanmoy Deb's fast nondominated sorting genetic algorithm with elite strategy (NSGA-II) is the most widely used one, and this research will adopt a multiobjective optimization algorithm based on NSGA-II.

The article "Robust Parameter Design for Cyclone System Based on Dual-Response Surface Method and Multiobjective Genetic Algorithm" was published in 2022. Journal: Comput Intell Neurosci.

## 4. The Double-Response Surface Method Proposed in This Paper

Although the double-response surface method solves the problems of lack of interaction items and lack of sequence of experiments in the process of robust design, the current research on double-response surface is mainly to analyze one quality characteristic, and now the products delivered to customers need to be comprehensively evaluated from the perspective of multiple dimensions and multiple quality characteristics. So, the robust parameter design of multiquality characteristics (response characteristics) has become an urgent problem to be solved, and the multiobjective genetic algorithm just provides the possibility for the realization of robust parameter design of multiresponse characteristics. The traditional optimization methods such as gradient descent method may fall into local extreme values, and the genetic algorithm has a strong ability in the global optimization problem and can solve the problem of local convergence.

For eye-type characteristic *Y*_1_, large-scale characteristic *Y*_2_ and small-scale characteristic *Y*_3_, the respective double-response optimization functions are as follows:

(5) $$\begin{array}{c} \text{min}F_{1}\left(x\right)=\omega_{Y_{1}\sigma }^{2}+{\left(\omega_{Y_{1}u}-\tau \right)}^{2},\\ \text{min}F_{2}\left(x\right)=\omega_{Y_{2}\sigma }^{2}+{\left(\frac{1}{\omega_{Y_{2}u}}\right)}^{2}\\ \text{min}F_{3}\left(x\right)=\omega_{Y_{3}\sigma }^{2}+\omega_{Y_{3}u}^{2}. \end{array}$$

Therefore, the multi response robust parameter optimization function based on the integration of multiobjective genetic algorithm and double response surface method is shown in formula (6).

(6) $$\begin{array}{c} \left\{\begin{array}{cc} \min & \left[F_{1}\left(x\right),F_{2}\left(x\right),F_{3}\left(x\right)\right],\\ \text{s.t}. & \left\{\begin{array}{c} lb\leq x\leq ub,\\ \text{Aeq}*x=\text{beq}\\ A*x\leq b, \end{array},\right. \end{array}\right. \end{array}$$

Moreover, for the acquisition of test data, the product table is used to design the test, and the response surface test design method is used for the inner table to ensure that the established model can reflect the changes of the surface and the influence of interaction terms. According to the two most unfavorable conditions, all the noise factors affecting the inner table test treatment are adopted the comprehensive error method. In other words, each treatment in the internal table runs once under each most unfavorable condition. Therefore, each test treatment will get two values, and the mean and standard deviation of these two values are used as the output response of this treatment.

The article "Robust Parameter Design for Cyclone System Based on Dual-Response Surface Method and Multiobjective Genetic Algorithm" was published in 2022. Journal: Comput Intell Neurosci.

## 5. Case Analysis

### 5.1. Background and Requirements of Test Design

The cyclone production system of a heavy medium coal preparation plant is a pressurized three product heavy medium cyclone production system, which is composed of two product heavy medium cyclone production systems in series. The first section is a high-density area, the products are gangue and medium clean coal, and the second section is a low-density area. Medium clean coal and some small particle size raw coal enter the system for screening, and the products are medium coal and clean coal. The schematic diagram of production process is shown in Figure 2. At present, domestic and foreign coal preparation enterprises adopt the method of “ensuring one end” for the quality control of coal preparation products, focusing on ensuring the quality of cleaned coal products. Coal quality indexes mainly include ash, calorific value, moisture, and so on. Since calorific value, moisture and other indexes can be derived from ash, clean coal ash is selected as the quality response characteristic of this study. In order to maximize the interests of the enterprise, the clean coal washing out rate, that is, the yield index, is also particularly important. Unilaterally meeting the low ash index may meet the requirements of external customers, but the clean coal yield will be greatly reduced, resulting in damage to the interests of the enterprise. Therefore, based on the recent customer demand and underground coal quality, the coal preparation plant decided to set the target of washed coal ash content of the coal preparation plant at 8.50% and the yield target at no less than 69.50% by carrying out the floating and sinking test of raw coal. The floating and sinking test results are shown in Table 1.

### 5.2. Test Design Scheme

In order to achieve the set response characteristic *y* and realize the stability of the system, it is necessary to determine the main controllable factors and noise factors affecting the response characteristics in the cyclone production system, that is, *x* and *u* in Figure 1, and reasonably set the value level of each factor in combination with the theory and practical experience of cyclone separation in heavy medium coal preparation plant. After consulting a large number of heavy medium coal preparation data [35], it is known that the cyclone production system includes three parameter types. One is the equipment structure parameters, such as the diameter of feed inlet and discharge outlet, and the other is the operating parameters, such as feed pressure and slime content. The other is fixed parameters, such as the washability of feed coal. Since the structural parameters of the equipment and the mechanism of coal are not determined by the production process, the following part will focus on the robust design of the operating parameters of the cyclone production system under the existing production conditions. Combined with relevant heavy medium coal preparation data, national and industrial standards, and with on-site management, the technicians decided to select the feed pressure (*x*_1_) in the low-density area, the solid-liquid ratio (*x*_2_) in the low-density area, the feed pressure (*x*_3_) in the high-density area and the suspended slurry content in the high-density area (*x*_4_) four parameters are used as important controllable factors, and the value level of each factor is set. Since the density of heavy medium will change in the separation process and cannot be controlled in a short time, two parameters of suspension density (*U*_1_) in low-density area and suspension density (*U*_2_) in high-density area are selected as noise factors, and the upper and lower deviations are allowed to be 5% respectively, as shown in Table 2.

The article "Robust Parameter Design for Cyclone System Based on Dual-Response Surface Method and Multiobjective Genetic Algorithm" was published in 2022. Journal: Comput Intell Neurosci.

The internal and external table method is used to design the test scheme. The response surface test design method is used to design the 4-factor 2-level test in the inner table. The center points in the test scheme are set as 6 and run 30 times in total. The surface is designed by the most unfavorable comprehensive error method, that is, each treatment in the internal table scheme runs once when the noise factor is the maximum value and the minimum value (one test). Therefore, the robust parameter design of the hydrocyclone production system requires a total of 60 tests. The test arrangement and test results are shown in Table 3, where 1 represents the high-level value, −1 represents the low-level value, and 0 is the central point value.

Neutralization in the table is the test results of ash characteristics under the two most unfavorable conditions, which is the mean value of the two test results, *σ*_*Y*_1_ is the standard deviation of the two most unfavorable cases and *σ*_*Y*_2_ is the test results and relevant statistical values of yield characteristics.

### 5.3. Robust Parameter Design of Cyclone Production System

#### 5.3.1. Model Fitting

According to the test design plan and test results, the double-response surface model including quadratic terms for ash characteristics and yield characteristics is established using the double-response surface method, and the effectiveness of the model is analyzed.

The article "Robust Parameter Design for Cyclone System Based on Dual-Response Surface Method and Multiobjective Genetic Algorithm" was published in 2022. Journal: Comput Intell Neurosci.

*Y*_1_ characteristics, the variance analysis results of the mean obtained by fitting analysis are shown in Table 4, and the estimated effects and coefficients are shown in Table 5.

It can be seen from Tables 4 and 5 that the *P* of the model is 0.02 < 0.05, so it is considered that the model is effective, and each estimated effect is significant. It is further verified that the residual error of the model meets the requirements, and there is no abnormality, as shown in Figure 3. Therefore, it can be considered that the fitting model of *u*_*y*1_ established is effective.

According to the aforementioned analysis, the fitting model of the mean value of *Y*_1_ characteristic is as follows:

(7) $$\begin{array}{c} U_{Y1}=8.4446+0.325x_{1}-0.05x_{2}+0.1029x_{1}^{2}. \end{array}$$

Similarly, the fitting models obtained are as follows:

(8) $$\begin{array}{c} \sigma_{Y1}=0.05436-0.00118x_{1}+0.00471x_{2}-0.00118x_{3}-0.00432x_{4}+0.0309x_{3}^{2}-0.0327x_{4}^{2}-0.02077x_{1}x_{2}+0.01724x_{1}x_{3}-0.02431x_{2}x_{3},\\ U_{Y2}=67.657+0.43x_{1}-0.45x_{2}-0.05x_{4}+1.615x_{4}^{2},\\ \sigma_{Y2}=1.225-0.068x_{1}-0.77x_{1}^{2}. \end{array}$$

According to the double-response surface method in part 2, the optimization functions are constructed for the mean and standard deviation models of *Y*_1_ and *Y*_2_ response characteristics respectively. The optimization function of *Y*_1_ (target type) is shown in formula (9). Since the model established by the model fitting part is obtained based on coding, the value range of controllable factor is [−1, 1]. Since *Y*_1_ is the target characteristic and is strictly not allowed to exceed the set standard by 8.50%.

(9) $$\begin{array}{c} \left\{\begin{array}{cc} \min & F_{1}\left(x\right)={\left(U_{Y1}-\tau \right)}^{2}+\sigma_{Y1}^{2},\\ s.t. & \left\{\begin{array}{c} -1\leq x_{i}\leq 1,i=1,2,3,4\\ U_{Y1}\leq 8.50\% \end{array}.\right. \end{array}\right. \end{array}$$

Similarly, the optimization function of *Y*_2_ characteristic (expected to be large) can be obtained as follows:

(10) $$\begin{array}{c} \min F_{2}\left(x\right)={\left(\frac{1}{U_{Y2}}\right)}^{2}+\sigma_{Y2}^{2}\\ \left\{\begin{array}{c} -1\leq x_{i}\leq 1,\;i=1,2,3,4\\ U_{Y2}\geq 69.5\% \end{array}.\right. \end{array}$$

According to the robust parameter design method integrating double-response surface and multiobjective genetic algorithm proposed in the third part of the paper, the optimization function of multiresponse characteristics can be obtained.

The number is as follows:

(11) $$\begin{array}{c} \min F_{1}\left(x\right)={\left(U_{Y1}-\tau \right)}^{2}+\sigma_{Y1}^{2},\\ \min F_{2}\left(x\right)={\left(\frac{1}{U_{Y2}}\right)}^{2}+\sigma_{Y2}^{2},\\ \left\{\begin{array}{c} -1\leq x_{i}\leq 1,i=1,2,3,4\\ U_{Y1}\leq 8.50\%\\ U_{Y2}\geq 69.5\% \end{array}.\right. \end{array}$$

Since the optimization function (11) includes nonlinear constraints, the external penalty function method is used to transfer the nonlinear inequality constraints to the objective function to obtain the final optimization function, as shown in formula (12), where *m* is a very large penalty coefficient, which is also the fitness function expression of multiobjective genetic algorithm.

(12) $$\begin{array}{c} \min F_{1}\left(x\right)={\left(U_{Y1}-\tau \right)}^{2}+\sigma_{Y1}^{2}+M*\min{\left(\left(8.50\%-U_{Y1}\right),0\right)}^{2},\\ \min F_{2}\left(x\right)={\left(1/U_{Y2}\right)}^{2}+\sigma_{Y2}^{2}+M*\min{\left(\left(U_{Y2}-69.5\%\right),0\right)}^{2},\\ \mathrm{s.t.}-1\leq x_{i}\leq 1,\;i=1,2,3,4. \end{array}$$

The parameters of the multiobjective genetic algorithm are set as follows: the optimal front-end individual coefficient Pareto fraction: 0.3, population size: 100, maximum iteration generations: 200, stop algebra limit: 200, fitness function value deviation function: 1*e* − 100. The obtained Pareto front-end distribution and the distance between individuals in the evolution process are shown in Figure 4.

The article "Robust Parameter Design for Cyclone System Based on Dual-Response Surface Method and Multiobjective Genetic Algorithm" was published in 2022. Journal: Comput Intell Neurosci.

According to the Pareto front-end distribution in Figure 4, the junction distribution is relatively uniform, indicating that the obtained solution is effective and the effect is good. Meanwhile, the other three subgraphs in the figure show that the distance and propagation speed between individuals are gradually decreasing, which indicates that with the increase of evolution, the diversity of the population gradually decreases and the solution gradually converges. Since the optimal front-end individual coefficient is 0.3 and the number of populations is 100, 30 groups of optimal solutions are obtained, of which 4 groups are close to or meet the requirements, as shown in Table 6.

As the *Y*_1_ characteristic is required to be strictly less than or equal to 8.50%, only the third group solution in Table 6 strictly meets the requirements. Therefore, the robust parameter design value (code value) of the hydrocyclone production system is (*X*_1_: 0.050332, *X*_2_: −0.772998, *X*_3_: −0.295515, *X*_4_: 0.999956), and the actual values are 150.50 kpa, 0.176143.52 kpa, and 30%, respectively. The optimal response characteristics that can be realized are *Y*_1_: 8.499% and *Y*_2_: 69.59%.

### 5.4. Comparative Analysis of the Effectiveness of the Method

The optimization function of each output characteristic established by the double-response surface method actually adopts the method of transforming constraints into objective functions, so as to transform them into unconstrained single-objective optimization problems. At present, most of the optimization functions with multiple output characteristics are transformed by the satisfaction function method. After transforming the multiobjective function into a single-objective function, the stability point of the system is obtained by derivation, the type of stability point is determined by canonical analysis, and the confidence interval of the optimal value is estimated according to the normal hypothesis. Therefore, this part shows the effectiveness and efficiency of this method by comparing the differences between the traditional optimization method and the proposed optimization method.

The article "Robust Parameter Design for Cyclone System Based on Dual-Response Surface Method and Multiobjective Genetic Algorithm" was published in 2022. Journal: Comput Intell Neurosci.

First, if each output characteristic optimizes its dual-response optimization function respectively, set the upper limit of *u*_*y*1_ to 8.500001%, the target to 8.50%, and the lower limit to 8.40%. The type is the desired type, and set *σ*_*Y*1_ is expected to be large. The response optimizer of Minitab is used to optimize the two functions at the same time. The results are shown in Figure 5.

Similarly, the lower limit of *u*_*y*2_ is set to 69.5%. In order to achieve large scale, the double-response optimization result of *Y*_2_ is obtained, as shown in Figure 6.

Considering two characteristics and four response functions at the same time, the results are shown in Figure 7, It can be seen from the figure that the distribution of two characteristics and four response function is relatively uniform, thus demonstrating the effectiveness of the proposed method. The optimization results of the proposed method and the aforementioned analysis results are summarized and Table 7 is obtained. It can be seen from the table that better output results can be obtained when a single output characteristic is optimized respectively. However, the calculated parameter value (factor values) are quite different, indicating that their respective optimizations cannot guarantee the overall optimization of the system. When considering two output characteristics at the same time, the traditional method is used to optimize four response functions at the same time. Although the standard deviation of *Y*_2_ characteristics is twice as small as that of the proposed method, the performance of the traditional method is not as good as that of the proposed method in the other three indexes, especially for *Y*_1_ ash characteristics, the optimization results are not only closer to the ash requirement of 8.50%, but also have less fluctuation, so as to ensure that the coal preparation plant has high process control ability. Moreover, the maximum yield obtained by the traditional method is 68.4146%, which does not meet the design requirement of 69.50% in the floating and sinking test. In conclusion, it can be seen that the method proposed in this study is better than the traditional multiresponse robust parameter design method as a whole.

The article "Robust Parameter Design for Cyclone System Based on Dual-Response Surface Method and Multiobjective Genetic Algorithm" was published in 2022. Journal: Comput Intell Neurosci.

## 6. Conclusion

This paper shows the feasibility of integrating double-response surface method and multiobjective genetic algorithm to solve the problem of robust parameter design under the condition of multiresponse characteristics of cyclone production system in heavy medium coal preparation plant is discussed. The conclusions are as follows: (1) the optimal value of response characteristic ash is 8.499%, the optimal value of yield is 69.59%, and the optimal controllable factors are 150.50 kpa, 0.176143.52 kpa, and 30%; (2) A double-response optimization model between response characteristics and influencing factors is established; (3) The effectiveness of double-response surface method and multiobjective genetic algorithm in the optimization process of production system of heavy medium coal preparation plant is verified, and the qualified and stable coal quality and maximum yield are realized; (4) It has changed the fire-fighting and passive quality management mode of coal preparation enterprises, and gradually changed to the preventive, autonomous, and stable quality management mode. The enterprises are no longer tired of dealing with the continuous coal quality problems, but realize the expected output by controlling the stability of influencing factors. When the whole system is gradually stable, the coal quality inspection link of coal preparation plant can even be cancelled or weakened; (5) Coal preparation enterprises are more confident to realize the accurate control of the production process. In conclusion, the proposed method can explore the relationship between system input and output, reduce the influence of noise on model output and determine the robust parameter values under the condition of multiresponse characteristics, thus providing scientific support for the transformation of quality management mode.

## Figures and Tables

**Figure 1:** Multi objective optimization problem.

**Figure 2:** Schematic diagram of cyclone production system in a heavy medium coal preparation plant.

**Figure 3:** Residual plot of *U*_*Y*1_ model.

**Figure 4:** Analysis diagram of multiobjective genetic algorithm.

**Figure 5:** Double-response optimization analysis diagram of *Y*_1_ characteristics.

**Figure 6:** Double-response optimization analysis of *Y*_2_ characteristics.

**Figure 7:** Optimization analysis of *Y*_1_ and *Y*_2_ response characteristics.

The article "Robust Parameter Design for Cyclone System Based on Dual-Response Surface Method and Multiobjective Genetic Algorithm" was published in 2022. Journal: Comput Intell Neurosci.

**Table 1:** Comprehensive table for float sink test of 50–0.5 mm raw coal.

Density level,kg/L%	Weight,kg	Productivity %		Ashcontent	Cumulative				
		The currentlevel	Totalsample		Floating object			Sediment	
					The currentlevel, %	Totalsample, %	Ashcontent, %	Productivity, %	Ash content, %
1	2	3	4	5	6	7	8	9	10
−1.30	0.52	7.40	6.07	3.61	7.40	6.07	3.61	100.00	20.27
1.30～1.40	4.41	62.73	51.46	7.19	70.13	57.53	6.81	92.60	21.60
1.40～1.50	0.75	10.67	8.75	13.57	80.80	66.28	7.70	29.87	51.85
1.50～1.60	0.19	2.70	2.22	22.85	83.50	68.49	8.19	19.20	73.12
1.60～1.80	0.09	1.28	1.05	34.01	84.78	69.54	8.58	16.50	81.36
+1.80	1.07	15.22	12.49	85.34	100.00	82.03	20.27	15.22	85.34

*Note.* Sampling location: 301 belts. Total weight of coal sample before floating and sinking: 8.60 kg, ash content: 21%. The red dotted line area focuses on the changes of the two response indicators.

**Table 2:** Controllable factor, noise factor, and factor value level.

Factor	Type	Level
*x*_1_	Controlled	140–160 kPa
*x*_2_	Controlled	1/6–1/4
*x*_3_	Controlled	140–150 kPa
*x*_4_	Controlled	20%–30%
*u*_1_	Uncontrollable	1.38–1.52 kg/cm^3^
*u*_2_	Uncontrollable	1.62–1.79 kg/cm^3^

**Table 3:** Experimental design scheme and test results.

Serial number	Point type	*x*_1_	*x*_2_	*x*_3_	*x*_4_	*Y*_11_	*Y*_12_	*Y*_21_	*Y*_22_	*U*_*Y*1_	*U*_*Y*2_	*σ*_*Y*1_	*σ*_*Y*2_
1	−1	0	0	0	−1	8.45	8.41	69.52	67.23	8.43	68.38	0.028284	1.619270
2	−1	0	0	−1	0	8.50	8.46	69.76	69.55	8.48	69.66	0.028284	0.148490
3	−1	0	−1	0	0	8.52	8.50	69.65	69.56	8.51	69.61	0.014142	0.063640
4	0	0	0	0	0	8.85	8.77	70.12	70.02	8.81	70.07	0.056569	0.070710
5	−1	0	0	0	1	8.50	8.52	69.44	69.57	8.51	69.51	0.014142	0.091920
6	−1	1	0	0	0	8.74	8.70	70.06	69.96	8.72	70.01	0.028284	0.070710
7	−1	0	1	0	0	8.35	8.42	65.44	67.28	8.39	66.36	0.049497	1.301080
8	−1	−1	0	0	0	8.29	8.33	63.25	64.22	8.31	63.74	0.028284	0.685890
9	0	0	0	0	0	8.47	8.32	68.87	64.21	8.40	66.54	0.106066	3.295120
10	−1	0	0	1	0	8.21	8.41	62.76	68.99	8.31	65.88	0.141421	4.405280
11	1	−1	−1	1	1	8.49	8.51	69.51	69.47	8.50	69.49	0.014142	0.028280
12	1	1	−1	−1	1	8.55	8.55	69.66	69.71	8.55	69.69	0.000000	0.035360
13	1	−1	1	−1	1	8.46	8.29	68.89	64.27	8.38	66.58	0.120208	3.266830
14	1	1	−1	−1	−1	8.40	8.51	67.78	69.55	8.46	68.67	0.077782	1.251580
15	1	1	−1	1	1	8.70	8.88	69.86	70.11	8.79	69.99	0.127279	0.176780
16	1	1	1	1	−1	8.50	8.54	69.51	69.62	8.52	69.57	0.028284	0.077780
17	1	−1	−1	1	−1	8.45	8.52	68.88	69.12	8.49	69.00	0.049497	0.169710
18	0	0	0	0	0	8.32	8.41	67.89	68.26	8.37	68.08	0.063640	0.261630
19	0	0	0	0	0	8.33	8.45	67.67	68.23	8.39	67.95	0.084853	0.395980
20	1	−1	−1	−1	1	8.65	8.72	69.99	70.05	8.69	70.02	0.049497	0.042430
21	1	1	1	1	1	8.52	8.54	69.51	69.64	8.53	69.58	0.014142	0.091920
22	0	0	0	0	0	8.35	8.41	67.45	66.53	8.38	66.99	0.042426	0.650540
23	1	−1	−1	−1	−1	8.71	8.72	69.94	69.97	8.72	69.96	0.007071	0.021210
24	1	−1	1	1	−1	8.51	8.55	69.52	69.61	8.53	69.57	0.028284	0.063640
25	1	1	−1	1	−1	8.57	8.67	69.77	69.87	8.62	69.82	0.070711	0.070710
26	1	1	1	−1	−1	8.47	8.54	68.25	69.63	8.51	68.94	0.049497	0.975810
27	0	0	0	0	0	8.32	8.42	65.32	68.71	8.37	67.02	0.070711	2.397090
28	1	1	1	−1	1	8.56	8.50	68.53	69.57	8.53	69.05	0.042426	0.735390
29	1	−1	1	1	1	8.55	8.52	69.55	69.47	8.54	69.51	0.021213	0.056570
30	1	−1	1	−1	−1	8.40	8.60	69.34	69.87	8.50	69.61	0.141421	0.374770

The article "Robust Parameter Design for Cyclone System Based on Dual-Response Surface Method and Multiobjective Genetic Algorithm" was published in 2022. Journal: Comput Intell Neurosci.

**Table 4:** Estimated effects and coefficients of *u*_*y*1_.

Term	Effect	Coefficient	Coefficient standard error	*T*	*P*
Constant		8.4446	0.0344	245.13	<0.001^*∗*^
*A*	0.6050	0.325	0.0101	1.02	0.038^*∗*^
*B*	−0.1000	−0.0500	0.0181	−1.78	0.047^*∗*^
*A∗A*	0.2058	0.1029	0.0445	2.31	0.029^*∗*^

*Note.* ^*∗*^ is significant. *S* = 0.0119337, R-Sq = 97.48%, R-Sq (adjustment) = 94.11%.

**Table 5:** Analysis of variance of *u*_*y*1_ fitting model.

Source	Freedom	Seq SS	Adj SS	Adj MS	*F*	*P*
Model	3	0.399350	0.399350	0.049919	88.09	0.002
Linear	2	0.226562	0.001765	0.107832	1.78	0.045
*A*	1	0.003306	0.003306	0.003306	5.83	0.045
*B*	1	0.223256	0.223256	0.223256	393.98	<0.001
Square	1	0.139194	0.139194	0.019885	35.09	0.007
*A∗A*	1	0.139194	0.139194	0.019885	35.09	0.007
Error	3	0.001531	0.001531	0.001531	2.70	0.199
Misfit	1	0.001700	0.001700	0.000567	0.064	0.001
Pure error	2	0.001700	0.001700	0.000567		

**Table 6:** Partial optimal solutions obtained by multiobjective genetic algorithm.

*x*_1_	*x*_2_	*x*_3_	*x*_4_	*U*_*Y*1_	*σ*_*Y*1_	*U*_*Y*2_	*σ*_*Y*2_
0.299078	−0.414492	0.008521	0.998234	8.571729	0.017855	69.531513	1.135788
0.262752	−0.621845	−0.235414	0.998063	8.568191	0.014995	69.608660	1.153973
0.050332	−0.772998	−0.295515	0.999956	8.499869	0.011689	69.591351	1.219627
0.352806	−0.421071	−0.274353	0.997759	8.593124	0.016355	69.556071	1.105166

**Table 7:** Comparative analysis.

Methods	*x*_1_	*x*_2_	*x*_3_	*x*_4_	*U*_*Y*1_	*σ*_*Y*1_	*U*_*Y*2_	*σ*_*Y*2_
Sole *Y*_1_	−0.5960	−0.7778	−0.1111	1.0	8.5007	0.0043	—	—
Sole *Y*_2_	1	−1	0	−1	—	—	70.1273	0.3873
Sole *Y*_1_, *Y*_2_	−1	1	1	1	8.4650	0.0322	68.4161	0.5233
Proposed method	0.050332	−0.772998	−0.295515	0.999956	8.499869	0.011689	69.591351	1.219627

## Data Availability

The data set can be accessed upon request.
